# A Method for Identifying Vesicle Transport Proteins Based on LibSVM and MRMD

**DOI:** 10.1155/2020/8926750

**Published:** 2020-10-19

**Authors:** Zhiyu Tao, Yanjuan Li, Zhixia Teng, Yuming Zhao

**Affiliations:** Information and Computer Engineering College, Northeast Forestry University, Harbin 150040, China

## Abstract

With the development of computer technology, many machine learning algorithms have been applied to the field of biology, forming the discipline of bioinformatics. Protein function prediction is a classic research topic in this subject area. Though many scholars have made achievements in identifying protein by different algorithms, they often extract a large number of feature types and use very complex classification methods to obtain little improvement in the classification effect, and this process is very time-consuming. In this research, we attempt to utilize as few features as possible to classify vesicular transportation proteins and to simultaneously obtain a comparative satisfactory classification result. We adopt CTDC which is a submethod of the method of composition, transition, and distribution (CTD) to extract only 39 features from each sequence, and LibSVM is used as the classification method. We use the SMOTE method to deal with the problem of dataset imbalance. There are 11619 protein sequences in our dataset. We selected 4428 sequences to train our classification model and selected other 1832 sequences from our dataset to test the classification effect and finally achieved an accuracy of 71.77%. After dimension reduction by MRMD, the accuracy is 72.16%.

## 1. Introduction

Protein, regarded as the material basis of life and the caretaker of life activities [1], participates in all the functions of maintaining individual survival, including catalyzing specific biochemical reactions and participating in immune response. The protein diversity is increased by alternative splicing and posttranslation modifications [2, 3]. Hence, the topic of protein function prediction came into being around the time of the birth of bioinformatics [4–11]. In view of the different functions of protein, there are various kinds to be classified [12–17]. Many scholars are devoted to the classification of different functions of an enzyme [18–23], and some apply themselves to the recognition of whether a protein sequence is an effecter protein. In this thesis, we attempt to determine if a protein is a vesicular transport protein.

Substances with small molecular weight, such as water or ions, will directly pass through the cell membrane by free diffusion or through the ion channels embedded in the cell membrane. However, macromolecular materials like proteins cannot directly pass through the cell membrane. In the process of transportation in and out of the cell, they are first surrounded by a layer of membrane generated by cell-forming vesicles and then through the fusion or rupture of vesicles with the cell membrane or various organelle membranes to complete material transportation. This process is called vesicular transport. The key role to facilitate this process is vesicular transporter, which is a kind of ubiquitous protein in the cell membrane and organelle membrane. When macromolecular materials are to be transported across the membrane, a specific vesicle transport will concentrate them or supervise the specific organelles to produce different vesicle structures to carry or to wrap the materials to be transmitted. Vesicle transport activity occurs widely between cells or within cells, such as the transmission of neurotransmitters between nerve cells and the operation of the immune system, which is essential for maintaining life. In the field of biology, there have been many advanced studies on cell vesicle transport, and the research areas are also diverse. For example, Rothman et al. [24] studied the problem about the transport of proteins in Golgi matrix, the composition, and structure of Golgi-coated vesicles. Liu et al. [25] concentrated on research about the effect vesicular transporter that plays in synaptic transmission and neurodegeneration. Similarly, many human diseases are also related to the abnormal action of vesicular transport in cells. Brain dopamine-serotonin vesicular transport disease, which can cause movement disorder in infancy, is closely related to vascular monoamine transporter 2 (VMAT2) [26]. In addition, many similar examples are constantly discovered. Increasingly, more diseases are associated with gene mutations, which are responsible for the vesicular transport function.

With the development of this field, an increasing number of vesicular transport proteins and other proteins have been found. There is growing desire for rapid identification of vesicular transporters, which is difficult to meet with biological technology. This type of research requires bioinformatics scholars to use machine learning and other computational methods to process and to analyze massive protein sequences. Thus far, the research on using computational methods to identify vesicle transporters is scant. In 2019, Le et al. [27] used PSSM matrix to store sequence features and convolutional neural network (CNN) to determine whether the sequence is a SNARE protein, which is a kind of vesicular transporter. In the same year, these authors used a classifier called GRU based on CNN to identify vesicular transporters. However, for the identification of protein, DNA and RNA, the process to deal with these problems is similar. In recent years, the two steps of the process, feature extraction and classification, have become increasingly complex, and this is also true in the field of identifying vesicular transporters. Meanwhile, we try as much as possible to use a simpler way of feature extraction and classification, to ensure a better classification effect. Finally, we use the composition descriptor in the composition, transition, and distribution (CTDC) and LibSVM as the methods of feature extraction and classification, which are widely used by many scholars. It is a novel idea about our research that the feature dimension of our final prediction process is reduced to 29. Our flowchart is shown in Figure 1.

## 2. Materials and Methods

### 2.1. Dataset

Our data come from the previous research of Le et al. These data have been processed by BLAST to ensure that the similarity between any two sequences is less than 30%. In addition, we use random undersampling in order to balance the number of positive and negative samples in the training set. Finally, there are 4428 sequences in the final training set and 1832 sequences in the test set.  Table 1 details the composition of the dataset.

### 2.2. Method to Feature Extraction

Feature extraction is very important for constructing a predictor [28–37]. We use the CTDC method in iLearn toolkit to extract features of protein sequences. Developed from iFeatures, iLearn is a comprehensive toolkit based on Python, which was designed by Chen et al. that can be downloaded at http://ilearn.erc.monash.edu. As a powerful platform, it not only integrates a series of feature extraction and analysis methods but provides many machine learning algorithms for classification. CTDC is the first part of the CTD feature method in iLearn based on the first of three descriptors.

CTD is a classic sequence feature extraction method that was first proposed by Dubchak et al. [38] in 1995. It consists of three descriptors: composition (C), transition (T), and distribution (D). Composition refers to the ratio of the number of single amino acids with specific properties (or several small amino acid sequence fragments with certain physical and chemical properties) in the whole sequence [39]. Composition can be expressed with the following formula:

(1) $$\begin{array}{c} \text{Composition}=\frac{n_{x}}{N}\left(x=a,b,c\cdots \right), \end{array}$$

where *x* represents amino acids with specific groups or sequence fragments with special physical and chemical properties, and *a*, *b*, and *c* represent different kinds of groups. *N* represents the total length of the sequence. The second descriptor represents the ratio of two closely adjacent groups to the total sequence calculated as

(2) $$\begin{array}{c} \text{transition}=\frac{yx+xy}{N-1}\left(x=a,b,c\cdots y=a,b,c\cdots \right). \end{array}$$

In Eq. (2), *xy* and *yx* denote two closely adjacent groups. The third descriptor, distribution, represents the general spreading state of special groups in the whole sequence. From the first amino acid of the sequence, calculate the proportion of an amino acid carrying a specific group in five subchains for all the amino acids in a sequence. These five chains contain the first, 25%, 50%, 75%, and 100% special amino acid from the first amino acid of the sequence.

After our experiment, the features extracted from transition and distribution contributed little to the classification effect, so we only select the features extracted from composition. In iLearn, there are 13 kinds of physicochemical properties adopted, and each physicochemical property has three kinds of amino acid combination patterns. The concrete meaning of these properties comes from the research results of Tomii and Kanehisa [40] in 1996.

### 2.3. Method for Classification

We use LibSVM method based on Weka. LibSVM is a library about the support vector machine (SVM) developed by Professor Lin et al. in 2001. It has been widely used in bioinformatics [41–54]. It has the advantages of being a small program that is flexible, with less inputting parameters, is open source to expand easily, and thus has become the most widely used SVM Library in China. This library tool can be accessed at https://www.csie.ntu.edu.tw/~cjlin/. Weka is a free and noncommercial mining platform, which has a series of functional modules that basically meet various needs in data analysis, such as a variety of different classification and regression algorithms and performing cross validation during classification, automatically. LibSVM classification has been supported since Weka version 3.5.

SVM is a kind of generalized linear classifier that relies on supervised learning [55–60]. The key to classification is to form a hyperplane in multidimensional feature space through algorithm calculation, which can approximate separate positive and negative samples; it can be expressed mathematically as

(3) $$\begin{array}{c} \omega^{T}X_{i}+b=0, \end{array}$$

In (3), *X* is a vector composed of coordinate values of any point on the hyperplane in each dimension and *ω* is a vector that we need to calculate. In addition, in order to make the sum of the distance between the positive and negative sample set and the hyperplane reach the farthest, we need to construct two planes parallel to the hyperplane as the interval boundary to distinguish the sample classification. However, in most cases, positive and negative samples cannot be completely divided on both sides of a plane, so generally we will allow some samples to be divided incorrectly, which we called soft interval. Finally, the problem is simplified to formula (4).

(4) $$\begin{array}{c} \underset{\omega ,b,\xi }{\min}\frac{1}{2}{\left\|\omega \right\|}^{2}+C\overset{m}{\underset{i=1}{\sum }}\xi_{i}s.t.y_{i}\left(\omega^{T}x_{i}+b\right)\geq 1-\xi_{i},i=1,2,\cdots ,m,\xi_{i}\geq 0, \end{array}$$

where *ξ*_*i*_ represents a relaxation variable for each sample point, and *C* is the penalty parameter that needs to be set manually according to the actual situation. The Lagrange function corresponding to formula (5) can be shown as

(5) $$\begin{array}{c} L\left(\omega ,b,\xi ,\alpha ,\beta \right)=\frac{1}{2}{\left\|\omega \right\|}^{2}+C\overset{m}{\underset{i=1}{\sum }}\xi_{i}+\overset{m}{\underset{i=1}{\sum }}\alpha_{i}\left[1-\xi_{i}-y_{i}\left(\omega^{T}x_{i}+b\right)\right]+\overset{m}{\underset{i=1}{\sum }}\beta_{i}\left(-\xi_{i}\right), \end{array}$$

where parameters *α*_*i*_ and *β*_*i*_ are Lagrange multipliers. At the same time, to solve the problem conveniently, we need to use the technique about Lagrangian duality and set the kernel function. The dual problem to Lagrange function is represented as

(6) $$\begin{array}{c} \underset{\alpha ,\beta }{\max}\underset{\omega ,b,\xi }{\min}L\left(\omega ,b,\xi ,\alpha ,\beta \right)\;s.t.\alpha_{\text{i}}\geq 0,\beta_{\text{i}}\geq 0\;i=1,2,\cdots ,m. \end{array}$$

In this experiment, the radial basis function (RBF) is adopted as the kernel function, which is also the default setting in LibSVM. Two parameters, the cost (*c*) and gamma (*g*), need to be determined before building the classification model by using Weka. The parameter *c* is called the penalty coefficient. The higher the value of *c* is, the easier it is to over fit. And *g* is a parameter of RBF function after it is selected as kernel which affects the speed of process of training and prediction. There is no universally recognized best method for parameter selection, and the common method is to let *c* and *g* take values within a certain range, and then set different *c* and *g* in the process of training set data classification. Finally, use cross validation to get the classification accuracy verified by the training set in this groups *c* and *g*, and select the group with the best classification result by comparison [61]. It is a complicated process, but in LibSVM toolkit, the parameter optimization is automated, and it no longer needs to be manually adjusted. We use the program, grid.py in the LibSVM tool folder to get the optimal parameters.

### 2.4. MRMD for Dimensionality Reduction

The max-relevance-max-distance (MRMD) is a dimensionality reduction algorithm, which was developed by Zou et al. [62, 63] in 2015 that can be downloaded at https://github.com/heshida01/mrmd/tree/master/mrmdjar. It is based on a series of distance functions to judge the feature independence. The process of dimensionality reduction consists of three steps. First, the contribution of each feature to classification is evaluated and then the contribution is quantified. Second, sort the features according to their contribution to the classification. Third, select different numbers of features in order to classify and then record the results. For example, select the first feature the first time, select the first two features the second time, etc., until the number of selected features reaches the maximum; that is, all features are selected, and the classification test stops. By comparing the results of these classification tests, the best group is selected, and the features selected in this group are retained and regarded as the result of dimension reduction.

MRMD algorithm analyzes the contribution of each feature to the prediction process mainly through two aspects, max relevance and max distance. Max relevance (MR) is used to calculate the Pearson correlation coefficient between features and samples to quantify the correlation between features and case classes. As shown in Formula (7), Pearson correlation coefficient is equal to the covariance divided by the product of their respective standard deviations.

(7) $$\begin{array}{c} \rho_{X,Y}=\frac{\mathrm{cov}\left(X,Y\right)}{\sigma_{X}\sigma_{Y}}. \end{array}$$

The vectors *X* and *Y* are composed of the *i*th feature from the sequence and the class label to which these sequences belong. Max distance (MD) is used to analyze the redundancy between features. Specifically, we calculate the three indexes between features:

(8) $$\begin{array}{c} \begin{array}{c} \text{ED}\left(X,Y\right)=\sqrt{\overset{N}{\underset{k=1}{\sum }}{\left(x_{k}-y_{k}\right)}^{2}},\\ \text{COS}\left(X,Y\right)=\frac{X\cdot Y}{\left\|X\right\|\cdot \left\|Y\right\|},\\ \text{TC}\left(X,Y\right)=\frac{X\cdot Y}{{\left\|X\right\|}^{2}+{\left\|Y\right\|}^{2}-X\cdot Y}. \end{array} \end{array}$$

In (8), these indexes are called Euclidean distance, Cosine similarity, and Tanimoto coefficient. The value of MD is obtained by comprehensive consideration of these three indexes.

Finally, the value of the contribution of the classification of each feature is obtained by adding the values of MR and MD in a certain proportion.

### 2.5. Evaluation of Classification Results

We adopt cross validation (CV) to evaluate the experimental results objectively. It is a classic, analytical method for judging the performance of a prediction model [64–78]. The core idea is to take out most of the samples in a given dataset to build a classification model, to leave a small part of the samples, to use the newly established model for prediction, and to calculate the forecast errors of these small samples and to record their sum of squares. This process continues until all samples are predicted once and only once. There are three common CV methods: hold-out method, K-fold cross validation (K-CV), and leave-one-out cross validation (LOO-CV). We take the second approach, K-CV.

In K-fold cross validation, the initial data are divided into k groups of subdatasets. A group of independent subdatasets are retained as the validation model data, and other k-1 subdatasets are used for training. In this way, we can get k models and take each prediction result of the classifier into account. In general, the operation is to take the average value of each index of every classification time from k models. The value of K can be set according to the actual situation, and here we set its value to 5. After 5-fold cross validation set in Weka, in order to evaluate the results of classification, some indexes are often used [79–85]. The metrics we use are recall, precision, MCC, and accuracy, and their corresponding formulas are as follows:

(9) $$\begin{array}{c} \begin{array}{c} \text{Recall}=\frac{TP}{TP+FN},\\ \text{Precision}=\frac{TP}{TP+FP},\\ \text{Accuracy}=\frac{TP+TN}{TP+FN+FP+FN},\\ \text{MCC}=\frac{1-\left(\left(FN/TP+FN\right)+\left(FP/TN+FP\right)\right)}{\sqrt{\left(1+\left(FP-FN/TP+FN\right)\right)\left(1+\left(FN-FP/TN+FP\right)\right)}}. \end{array} \end{array}$$

For the convenience of description, we use “positive” to represent vesicular transporters and “negative” to represent nonvesicular transporters. In (7), the letter *T* means true (correct). The letter *N* means false (incorrect). *P* is the positive sample, and *N* represents the negative sample. For example, *TP* means that the positive samples are correctly identified.

## 3. Results and Discussion

After optimizing the parameters of the dataset having the whole 39 dimensional features extracted by CTDC, we first implement classification without dimension reduction operation. By using the parameter optimization function in LibSVM, we can automatically find the most suitable *c* and *g*; finally, the value of *c* is 2048 and *g* is 0.5. The classification accuracy of train set is 66.84% by Weka. For a total of 4428 samples, 653 positive samples and 815 negative samples are misclassified. For test set, the accuracy reaches 71.77%. For 1832 samples, there are 94 positive samples and 416 negative samples that are misclassified.

Simultaneously, we also test the datasets, which are processed by dimension reduction to judge the effect of MRMD method dimension reduction on classification results. First, we use MRMD for training set. After dimension reduction, the sample space dimension is reduced from 39 to 21. Second, we leave the feature of the test set selected by MRMD in training set and delete the others. Then, we do the same operation for the reduced dimension dataset. The optimal parameters *c* and *g* are 128 and 2, respectively. The classified accuracy of training set is 66.96% and test set is 72.16%. In train set, 656 positive samples and 807 negative samples are misclassified. In test set, 94 positive samples and 416 negative samples are misclassified.

To show more vividly the number of samples that have not been dimensionally reduced and have been correctly predicted, we have drawn Figure 2. *TP* represents the vesicle transporters predicted correctly, and *TN* is regarded as the nonvesicular transporters predicted incorrectly. From Figure 2, we can clearly see that the number of correctly predicted samples after dimensionality reduction is basically the same as that without dimensionality reduction. However, from another point of view, although this technique cannot classify more samples, correctly, it eliminates some features that do not contribute much to the classification and reduces the complexity of the classification process.

Of course, if it is unreasonable and incomplete to judge the prediction effect only by the accuracy rate, we need to know other indicators about the classification results to evaluate the result more objectively. For this reason, we list the four indexes, recall, precision, accuracy, and MCC, in the performance of classification of reduced dimension and not reduced dimension and create Table 2 to represent it.

In Table 2, it is obvious that the prediction results using the 21 features after dimensionality reduction have not decreased. This proves that MRMD has no negative effect on the prediction. In addition, because MRMD calculates the contribution of each feature to classification and sorts them in the process of dimensionality reduction, we can understand which features have great differences between vesicular transporters and nonvesicular transporters. For example, according to the calculation of MRMD, the 32nd feature, called charge. G2, is ranked first after dimensionality reduction, which indicates that this feature has the greatest difference between positive and negative samples. The 13th feature, the hydrophobicity_CASG920101.G1, is in second place, which means that the degree of difference between two categories is second only to the 32nd feature and so on. The specific meaning of these characteristics can be found in chapter 2.2 of Tomii et al.: they represent different states of physical and chemical properties, such as hydrophobicity, normalized van der Waals volume, polarization, and polarizability. This partly explains whether a protein becomes a vesicle transporter because some amino acid combinations in their sequences appear physical and possess chemical properties that other proteins do not. Certainly, these are not the only factors that determine protein function.

## 4. Conclusion

At present, in protein classification, scholars often extract a large number of features or the classification methods used are very complex. In our research, we used CTDC feature extraction combined with MRMD feature screening and dimensionality reduction. It is worth mentioning that the MRMD adopted to reduce the dimension, which not only reduces the number of features used in classification, but also has no negative interference to the prediction effect. Finally, we used only 21 features to complete the prediction of vesicle transporters and achieved a satisfactory result. The accuracy of our prediction method is 66% for training set by 5-fold cross validation and 72% for test set after dimension reduction. Compared with the widely used convolution neural network (CNN) or deep neural network (DNN), although it will obtain higher accuracy, there are also problems of over fitting and poor interpretability of classification process. The operation process of these methods cannot be explained, and each parameter in the classifier is adjusted by negative feedback according to the actual and theoretical results. The prediction process relies on the mutual accumulation of input and output of a series of individual neurons. It is difficult to say whether the result is related to the specific amino acid arrangement or some specific groups. However, for these classical characteristics, the sequence feature often means that there are some rules in the arrangement of amino acids in the sequence. It may be helpful for scholars to judge whether an unknown protein is a vesicular transporter. Through our study, the difference degree of each feature between positive and negative samples differs according to the calculation of MRMD. The features, like charge. G2 and hydrophobicity_Casg920101.G1, ranked first and second, respectively, and indicate that these physicochemical properties play a key role in the recognition of vesicle transporters. Moreover, the best classification results can be obtained by selecting the first 21 features, which also indicates that the content of amino acid combinations of the remaining 18 features represented between vesicular transporter and nonvesicular transporter is not significantly different. The difference in the content of these groups with specific physicochemical properties also helps to explain why proteins exhibit specific functions.

## Figures and Tables

**Figure 1:** Flowchart of identifying vesicular transporters.

**Figure 2:** Number of samples correctly predicted.

**Table 1:** The dataset used in this study.

	Original	Original train set	Train set	Test set
Vesicular transport	2533	2214	2214	319
Nonvesicular transport	9086	7573	2214	1513

**Table 2:** Comparison of classification results.

	Recall	Precision	Accuracy	MCC
39 characteristics	0.718	68.65%	71.77%	0.327
21 characteristics	0.722	70.53%	72.16%	0.342

## Data Availability

Experimental data can be obtained from https://github.com/taozhy/identifying-vesicle-transport-proteins or ask the author directly by email: 1765145064@qq.com.
